This article has been retracted.

# Protective effects of calorie restriction and 17-β estradiol on cardiac hypertrophy in ovariectomized obese rats

**DOI:** 10.1371/journal.pone.0282089

**Published:** 2023-04-25

**Authors:** Zahra Hajializadeh, Mohammad Khaksari, Shahriar Dabiri, Fatemeh Darvishzadeh Mahani, Alireza Raji-Amirhasani, Mohammad Abbas Bejeshk

**Affiliations:** 1 Physiology Research Center, Institute of Neuropharmacology, Kerman University of Medical Sciences, Kerman, Iran; 2 Endocrinology and Metabolism Research Center, Institute of Basic and Clinical Physiology Sciences, Kerman University of Medical Sciences Kerman, Kerman, Iran; 3 Pathology and Stem Cell Research Center, Kerman University of Medical Sciences, Kerman, Iran; 4 Department of Physiology and Pharmacology, Afzalipour Faculty of Medicine, Kerman University of Medical Sciences, Kerman, Iran; Universidade Federal do Rio de Janeiro, BRAZIL

## Abstract

Obesity and menopause lead to cardiovascular diseases. Calorie restriction (CR) can modulate estrogen deficiency and obesity-related cardiovascular diseases. The protective effects of CR and estradiol on cardiac hypertrophy in ovariectomized obese rats were explored in this study. The adult female Wistar rats were divided into sham and ovariectomized (OVX) groups that received a high-fat diet (60% HFD) or standard diet (SD) or 30% CR for 16 weeks, and then, 1mg/kg E2 (17-β estradiol) was injected intraperitoneally every 4 days for four weeks in OVX-rats. Hemodynamic parameters were evaluated before and after each diet. Heart tissues were collected for biochemical, histological, and molecular analysis. HFD consumption led to weight gain in sham and OVX rats. In contrast, CR and E2 led to body weight loss in these animals. Also, heart weight (HW), heart weight/body weight (HW/BW) ratio, and left ventricular weight (LVW) were enhanced in OVX rats that received SD and HFD. E2 reduced these indexes in both diet conditions but reduction effects of CR were seen only in HFD groups. HFD and SD feeding increased hemodynamic parameters, ANP (atrial natriuretic peptide) mRNA expression, and TGF-β1(transforming growth factor-beta 1) protein level in the OVX animals, while CR and E2 reduced these factors. Cardiomyocyte diameter and hydroxyproline content were increased in the OVX-HFD groups. Nevertheless, CR and E2 decreased these indicators. The results showed that CR and E2 treatment reduced obesity-induced-cardiac hypertrophy in ovariectomized groups (20% and 24% respectively). CR appears to have almost as reducing effects as estrogen therapy on cardiac hypertrophy. The findings suggest that CR can be considered a therapeutic candidate for postmenopausal cardiovascular disease.

## Introduction

Obesity is a significant challenge in developing countries because it represents the main risk for diet-related chronic diseases like cardiovascular disease (CVD) [1]. CVD is the leading cause of death in women which occurs mostly in postmenopausal women [2]. Also, 65% of high blood pressure in women is directly attributed to weight gain and obesity [3]. High blood pressure often leads to cardiac hypertrophy, which is a crucial risk factor for heart failure development [4]. The patterns of cardiac hypertrophy are different in men and women [5]. Cardiac hypertrophy incidence in postmenopausal women is more than in age-matched men [6]. In fact, estrogen deficiency causes developmental events that lead to cardiac hypertrophy [7]. Various studies have shown that estrogen reduces hypertension and prevents cardiac hypertrophy [7–9]. Also, it has been revealed that estrogen therapy decreased cardio-metabolic risk factors such as LDL, cholesterol, insulin, and glucose levels in postmenopausal women and rats [10, 11]. Hormone-replacement therapy may alter the risk of CVD by several mechanisms such as alterations in plasma concentrations of glucose, insulin, hemostatic factors, and blood pressure [11].

Also, obesity impairs the natriuretic responses. Therefore, the deficit in the natriuretic peptide system leads to obesity-related hypertension [12]. Atrial natriuretic peptide (ANP) is a peptide hormone often released in response to mechanical stretch through atrial cardiomyocytes [13]. ANP has been shown to be involved in the regulation of blood volume and blood pressure [14]. Furthermore, ANP plays an important autocrine role as a cardiac hypertrophy inhibitor and is also a direct cellular growth moderator [15]. However, impairment in the expression of the ANP gene leads to cardiac hypertrophy [16]. Female steroid hormones affect the cardiac natriuretic hormone system. A progressive reduction in ANP has been observed after the menopausal condition [17]. It has been revealed that E2 increased ventricular ANP gene expression in spontaneously hypertensive rats [18].

Obesity leads to undergoing cellular and molecular alterations in adipose tissue that affect systemic metabolism and produce several pro-inflammatory factors that might be contributing to the occurrence of cardiovascular complications [19]. Transforming growth factor beta (TGF-β) is one of the profibrotic cytokines and crucial mediators of cardiac fibrosis that induces fibroblast proliferation, cardiomyocyte hypertrophy, and fibrosis. It has been shown that inhibition of TGF-β signaling reduces fibrosis and prevents cardiac dysfunction in various models of maladaptive cardiac remodeling [20, 21], whiles TGF-β overexpression has been revealed to induce cardiac hypertrophy in transgenic mice [22]. It has been demonstrated that several cardiac hypertrophic pathways that are stimulated via TGF-β are regulated by ANP [23, 24]. Also, it has been reported that estrogen deficiency leads to the elevation of TGF-β and as result pathological cardiac remodeling [25].

As mentioned above, obesity is a significant contributor to CVD prevalence and increased morbidity and mortality. It is apparent that alterations in feeding habits through diets can be effective. Among different diets, calorie restriction (CR) as a non-pharmacological approach, has obtained popularity for its protective effects on numerous organs [26]. It has been revealed that moderate CR has a protective effect against the development of CVD, hypertension, and obesity in humans [27]. A study has reported that intermittent and continuous restrictive diets lead to cardio-metabolic health in obese postmenopausal women [10]. Moreover, it has been indicated that a combination of intermittent fasting with CR is effective for body weight loss and cardioprotection in women with obesity [28]. Also, it has been revealed that CR diminished ANP gene expression in rats [29]. In obese men, weight loss reduced blood pressure, and elevation in ANP can contribute to blood pressure decrement in obese individuals [30].

According to the role of CR and E2 in the prevention and treatment of CVD, and since the interaction of the E2 and dietary intervention programs in obesity-induced cardiac hypertrophy in postmenopausal conditions has not yet been fully clarified, therefore, the aim of the present study was to investigate the effects of CR or E2 on obesity-induced cardiac hypertrophy in the animal postmenopausal model and reveal some relevant mechanisms. Whether CR would result in the improvement of cardiovascular injuries induced by obesity in postmenopausal conditions. To answer this question, molecular and histopathology methods, and non-invasive evaluation of hemodynamic parameters were used in an animal menopause model.

## Materials and methods

### Animals

Female Wistar rats weighing 200–250 g were obtained from the Animal Center of Kerman University of Medical Sciences, Kerman, Iran. The animals (3 per cage) were maintained under controlled temperature conditions (23 ±3°C) and light (from 07:00 to 19:00 h) and had free access to water and standard chow. The study was accepted by the “Ethics Committee in Animal Experimentation of Kerman University (No: IR.KMU.REC.1399.566)” and performed based on the recommendations of the National Institutes of Health Guide for the Care and Use of Laboratory Animals.

### Experimental groups and diet protocols

As shown in Fig 1, rats were randomly divided into two main sham-operated and OVX groups as follows:

1. Sham-operated groups: the animals were maintained on a standard diet (SD) [30% fat, 55% carbohydrate, and 15% protein] for 16 weeks (Sham+SD, n = 7); Sham-operated animals were maintained on a 60% high-fat diet (HFD) [60% fat, 15% carbohydrate and 25% protein] for 16 weeks (Sham+HFD, n = 7); Sham-operated animals were maintained on SD (8 weeks) and then underwent food restriction (calorie restriction: CR; 70% daily food of Sham+SD group) for 8 weeks (Sham+SD+CR, n = 7); Sham-operated animals were maintained on HFD (8 weeks) and then underwent CR (70% daily food of Sham+HFD group) for 8 weeks (Sham+HFD+CR, n = 7).
2. OVX groups: ovariectomized rats were subdivided in a similar pattern to the sham groups [(OVX+SD, OVX+HFD, OVX+SD+CR, OVX+HFD+CR). At the end of 16 weeks, to assess the effects of E2 on cardiac hypertrophy the OVX animals were divided into 8 groups, randomly. OVX+SD rats treated with E2 for 4 weeks (OVX+SD+E2, n = 7); 2) OVX+HFD rats treated with E2 for 4 weeks (OVX+HFD+E2, n = 7); 3) OVX+SD+CR rats treated with E2 for 4 weeks (OVX+SD+CR+E2, n = 7); 4) OVX+HFD+CR rats treated with E2 for 4 weeks (OVX+HFD+CR+E2, n = 7), Oil (solvent of E2) groups: OVX rats were classified in a similar pattern as the E2-treated groups (OVX+SD+Oil, OVX+HFD+Oil, OVX +SD+CR+Oil, OVX+HFD+CR+Oil). In order to imitate the natural estrous cycle, E2 (1 mg/kg) [31] and sesame oil (solvent of E2) were injected every four days intraperitoneally (i.p.) for 4 weeks. Also, during four weeks of treatment, animals were placed on the SD [32].

**Fig 1:** Schematic of A) animal classification, B, and C) time tables of the experimental protocol. OVX: Ovariectomy, SD: Standard diet, HFD: High-fat diet, CR: Calorie restriction, E2: 17-β Estradiol, Oil: Sesame oil.

### Bilateral ovariectomy

The animals were anesthetized with a dose of 80/10 mg/kg ketamine and xylazine intraperitoneally (Alfasan Co., Utrecht, Netherlands). A tiny longitudinal cutting was made in the stomach and then skin and abdominal muscles were opened, and ovaries were resected. After that, 1–2 ml of sterile normal saline was poured into the abdomen, and the skin was sutured. In the sham surgery, an analogous incision was made, yet the ovaries were not resected. The experiments were carried out 2 weeks after OVX [33].

### Induction of dietary obesity

In animals, obesity was induced by feeding a 60% high-fat diet [(HFD): 60% fat, 15% carbohydrate, and 25% protein] for 16 weeks (Royan Institute, Isfahan, Iran).

### Calculation of meal size and calorie restriction (CR)

The one-week food intake amount was measured in the sham animals to specify the meal size in the CR groups. The animals had access to the food (standard or high fat) freely, and the average daily intake was evaluated. Then, 70% of the total daily consumption of the group that had free access to food was calculated and given to the CR group for 8 weeks [34].

### Experimental procedures

The body weight of rats was measured weekly. At baseline, before and after each diet in the entire study period, hemodynamic parameters were measured. At the end of the study, rats were anesthetized by exposed to a CO2 atmosphere and decapitated and then heart tissues were removed, weighed, and used for further analysis of histology, determination of hydroxyproline levels, and gene expression (4 hearts/group for each of the 3 techniques). TFG-β1 (Transforming growth factor beta 1) was measured using the ELISA method and also RNA extraction and real-time polymerase chain reaction (Real-time PCR) were carried out for determining the gene expression of ANP (atrial natriuretic peptide) in the left ventricles (LVs).

### Hemodynamic parameters measurement

The hemodynamic parameters were recorded with the tail-cuff method on an LE5002 non-invasive blood pressure system (Panlab Harvard Apparatus, Australia) on the baseline, before and after each diet. The animal tail was placed in contact with a cuff, and a pulse transducer was used to measure the systolic blood pressure (SBP), diastolic blood pressure (DBP), heart rate (HR), and mean arterial pressure (MAP). An average of 4 pressure readings was recorded for each measurement [35].

### TGF-β1 measurement

First LV heart tissues were removed and placed in ice-cold saline. Afterward, tissues were homogenized and centrifuged for 10 minutes at 1000 rpm, and finally, the supernatant was separated. Then, the level of TGF-β1 in LV heart tissues was measured using the ELISA method according to the kit instructions (Cat.No: ab119558, Abcam, MA, USA) [36].

### Histological analysis for cardiomyocyte diameter measurement

Heart tissues were fixed in 10% buffered formaldehyde and then embedded in paraffin. Cross sections (4μm thick) of the LV were stained with hematoxylin and eosin stain (H&E) and observed under a light microscope (Nikon Labophot, Japan). Cardiomyocyte diameters were measured by two investigators who were blind to the animal groups. In each sample, approximately 50 cardiomyocytes from the LV were examined, and the cardiomyocyte diameters were measured. The mean value of 50 measurements indicated one sample [1].

### Hydroxyproline assay

In the biochemical assessment, hydroxyproline in the left ventricle as an index of tissue collagen contents was measured by a commercial kit (Kiazist, Iran) as described in its protocol manual. First, the samples of rat cardiac LV were homogenized and digested in 12M HCl and then the supernatant turns an orange-purple color following an oxidation reaction with a chromogen. Finally, colorimetric outcomes were read by Bio-Rad Microplate Reader at a wavelength of 550 nm [37].

### RNA extraction and real time-PCR

Total RNA was extracted from heart tissues via a commercial RNA synthesis kit based on the manufacturer’s instructions (Kiazist, Iran). The purity and concentration of the RNA were assessed by measuring the absorbance at 260 and 280 nm wavelengths. An equal amount of RNAs (1μg) was used for cDNA synthesis (cDNA synthesis kit, Kiazist, Iran). Then, for real-time PCR, cDNA (2 μL), forward primer (2 μL), and reverse primer (2 μL) of each gene [*ANP* and *Actb* (as a housekeeping gene)] were added to 10 μL of SYBR® Green real-Time Master Mix. Then, the amount of gene expression was measured with System Step One™ real-Time PCR (ABI 1 plus, USA). Differences in each target gene expression were measured relative to the values of *Actb* (as a housekeeping gene) by the 2^–ΔΔCt^ method [38]. The primer sequences used for real-time PCR were:

*ANP* forward: 5′GAGCGAGCAGACCGATGAA3′

*ANP* reverse: 5′GTCAATCCTACCCCCGAAGC3′

*Actb* forward: 5′CCCGCGAGTACAACCTTCTT3′

*Actb* reverse: 5′CCATACCCACCATCACACCC3′

### Statistical analysis

Data were expressed as mean ± SEM and analyzed using GraphPad Prism 6 software. Data were analyzed using one-way ANOVA for body weight changes (%), heart weight, heart weight/body weight ratio, left ventricular weight, hemodynamic parameters (in E2-treated groups), cardiomyocyte diameter, hydroxyproline content, *ANP* mRNA expression, and TGF-β1 protein level followed by a Tukey post-hoc test. Two-way ANOVA was used for hemodynamic parameters (at baseline, before and after each diet) followed by Tukey post-hoc test. Data were considered statistically significant at the p<0.05 level.

## Results

### The effect of CR on body weight and heart weight changes

The body weight changes (%), heart weight (HW), heart weight/body weight (HW/BW) ratio, and left ventricular weight (LVW) were measured in sham and OVX groups after feeding with HFD or SD (Table 1). The initial body weight of the animals was measured on the first day of the experiment (before diet administration) and the final body weight at the end of the sixteenth week. OVX+SD and OVX+HFD groups showed more body weight gain (38.46% and 66.85%, respectively) than Sham+SD and Sham+HFD groups. Also, the body weight in the Sham+HFD group was more than the Sham+SD group (P<0.05). On the other hand, CR led to body weight loss in sham and OVX groups that received SD (P<0.001) and HFD (P<0.001) compared to before each diet. The values of HW, HW/BW ratio, and LVW in OVX+SD (P<0.001, P<0.01, and P<0.05, respectively) and OVX+HFD (P<0.001, P<0.01, and P<0.001, respectively) groups, were more than Sham+SD and Sham+HFD groups. In contrast, HW (P<0.05), HW/BW ratio (P<0.01), and LVW (P<0.001) in OVX+HFD+CR groups were less than before the diet. There were no significant changes in the HW, HW/BW ratio, and LVW with or without CR between the Sham groups.

**Table 1:** Comparison of CR effects on body weight changes, HW, HW/BW ratio, and LVW in Sham and OVX rats.

Parameters	Sham				OVX			
	SD	HFD	SD+CR	HFD+CR	SD	HFD	SD+CR	HFD+CR
**Body weight changes (%)**		*	***	+++	**	+++ ###	### †	&&& **^**
	27.27±1.78	35.27±1.45	-5.23±1.18	-1.57±1.09	38.46±2.22	66.85±2.32	-1.63±0.99	11.41±3.03
**HW (mg)**								
					***	+++ #	# † ≌	& **^^**
	0.63±0.02	0.75±0.06	0.57±0.05	0.62±0.04	0.92±0.02	1.14±0.08	0.70±0.02	0.89±0.02
**HW/BW ratio (⊆10** ^**−3**^ **)**	3.40±0.15	3.77±0.23	3.06±0.19	3.10±0.11	**	++ #	## ≌† ≌	&& **^^^**
					4.54±0.23	5.60±0.26	3.11±0.16	4.27±0.24
**LVW (mg)**	0.47±0.03	0.65±0.05	0.49±0.06	0.51±0.03	*	+++ #	# †	&&& **^**
					0.79±0.02	0.92±0.02	0.51±0.03	0.72±0.03

Data are expressed as mean ± SEM, n = 7 rats/group. ***P<0.001, **P<0.01 and *P<0.05 *VS*. Sham+SD; ^+++^P<0.001 and ^++^P<0.01 *VS*. Sham+HFD, ^###^P<0.001, ^##^P<0.01 and ^##^P<0.05 *VS*. OVX+SD; ^&&&^P<0.001, ^&&^P<0.01 and ^&^P<0.05 *VS*. OVX+HFD; ^†^ ≌P< 0.05 *VS*. Sham+SD+CR; ^^^^^P<0.001, ^^^^P<0.01 and ^^^^P<0.05 *VS*. Sham+HFD+CR. HW: Heart weight, BW: Body weight, LVW: Left ventricular weight, HFD: High-fat diet, SD: Standard diet, CR: Calorie restriction, Sham: Ovary-intact, OVX: Ovariectomy

### The effect of E2 treatment on body weight and heart weight changes

As shown in Table 2, BW, HW, HW/BW ratio, and LVW in OVX+SD+E2 (P<0.001, P<0.001, P<0.01, P<0.01, respectively) and OVX+HFD+E2 (P<0.001) groups were less than OVX+SD+Oil and OVX+HFD+Oil groups. Also, E2 diminished BW (P<0.001), HW (P<0.05, P<0.001), HW/BW ratio (P<0.05, P<0.001), and LVW (P<0.05) in SD+CR and HFD+CR groups more than the SD+CR+Oil and HFD+CR+Oil groups. The effects of E2 on BW (P<0.001), HW (P<0.05), HW/BW ratio (P<0.05), and LVW (P<0.05) reduction in the SD+CR group were more than the other groups.

**Table 2:** Effects of E2 treatment on body weight changes, HW, HW/BW ratio, and LVW in OVX rats.

Parameters	Oil				E2			
		SD	HFD	SD+CR	HFD+CR	SD	HFD	SD+CR	HFD+CR
**Body weight**					***	+++	#	&&&
**changes (%)**	13.06±1.27	20.42±2.01	6.21±0.94	13.49±2.23	9.38±0.97	-5.67±0.95	-15.61±0.66	14.91±1.19
**HW (mg)**	0.93±0.01	1.16±0.08	0.72±0.02	0.91±0.02				
						***	+++	#	&&&
						0.70±0.02	0.72±0.06	0.50±0.02	0.61±0.04
**HW/BW ratio (⊆10** ^**−3**^ **)**	4.90±0.30	6.05±0.29	3.64±0.15	4.63±0.24	**	+++	#	&&&
					3.40±0.17	3.67±0.22	2.57±0.15	3.09±0.11
**LVW (mg)**	0.78±0.02	1.09±0.08	0.67±0.02	0.72±0.03	**	+++	#	&
					0.58±0.05	0.65±0.05	0.46±0.03	0.50±0.01

Data are expressed as mean ± SEM, n = 7 rats/group. ***P<0.001 and **P<0.01 *VS* SD+Oil; ^+++^P<0.001 *VS* HFD+Oil; ^#^P<0.05 *VS* SD+CR+Oil; ^&&&^P<0.001 and ^&^P<0.05 *VS* HFD+CR+Oil. HW: Heart weight, BW: Body weight, LVW: Left ventricular weight, HFD: High-fat diet, SD: Standard diet, CR: Calorie restriction, E2: 17-β estradiol, Oil: Sesame oil

### The effect of CR on hemodynamic parameters

OVX+HFD groups revealed higher MAP, SBP, DBP, and HR values in the 2nd (P<0.01) and 4th (P<0.001) months than Sham+HFD groups. (Fig 2A–2D). Also, MAP, SBP, DBP, and HR values in 2nd (P<0.01, P<0.05, P<0.01, P<0.01; respectively) and 4th (P<0.01) months, in OVX+SD groups, were more than the Sham+SD groups. In contrast, MAP, SBP, DBP, and HR values in OVX+SD (P<0.05, P<0.001, P<0.01, P<0.001, respectively) and OVX+HFD (P<0.01) groups were lower than before each diet. No significant differences in the hemodynamic data were observed with or without CR between the Sham groups.

**Fig 2:** Effects of CR on hemodynamic parameters. Data are expressed as mean ± SEM (n = 7 rats/group). A: MAP (mmHg), B: SBP (mmHg), C: DBP (mmHg), and D: HR (bpm). ***P<0.001, **P<0.01 and *P<0.05 *VS*. Sham+SD; ^+++^P<0.001 and ^++^P<0.01 *VS*. Sham+HFD; ^###^P<0.001, ^##^P<0.01 and ^#^P<0.05 *VS*. OVX+SD; ^&&^P<0.01 *VS*. OVX+HFD; ^†^P<0.05 *VS*. Sham+SD+CR; ^^^^^P<0.001, ^^^^P<0.01 and ^^^P<0.05 *VS*. Sham+HFD+CR. CR: Calorie restriction, HFD: High-fat diet, SD: Standard diet, MAP: Mean arterial pressure, SBP: Systolic blood pressure, DBP: Diastolic blood pressure, HR: Heart rate, Sham: Ovary-intact, OVX: Ovariectomy.

### The effect of E2 treatment on hemodynamic parameters

As shown in Fig 3A–3D, E2 administration displayed more reduction in MAP, SBP, DBP, and HR values in OVX+SD (P<0.05) and OVX+HFD (P<0.01) groups than in OVX+SD+Oil and OVX+HFD+Oil groups. Also, E2 attenuated these indexes in SD+CR (P<0.05) and HFD+CR (P<0.01, P<0.01, P<0.05, and P<0.001, respectively) groups more than SD+CR+Oil and HFD+CR+Oil groups.

**Fig 3:** Effects of E2 administration on hemodynamic parameters in OVX rats. Data are expressed as mean ± SEM (n = 7 rats/group). A: MAP (mmHg), B: SBP (mmHg), C: DBP (mmHg), and D: HR (bpm). *P<0.05 *VS*. SD+Oil; ^++^P<0.01 *VS*. HFD+Oil; ^###^P<0.001 and ^#^P<0.05 *VS*. SD+CR+Oil; ^&&&^P<0.001, ^&&^P<0.01 and ^&^P<0.05 *VS*. HFD+CR+Oil. CR: Calorie restriction, HFD: High-fat diet, SD: Standard diet, MAP: Mean arterial pressure, SBP: Systolic blood pressure, DBP: Diastolic blood pressure, HR: Heart rate, OVX: Ovariectomy, E2: 17-β estradiol, Oil: Sesame oil.

### The effect of CR on TGF-β1 level

As shown in Fig 4, OVX+SD and OVX+HFD groups had higher protein levels of TGF-β1 than Sham+SD and Sham+HFD groups (P<0.001). On the other hand, TGF-β1 protein levels in OVX+SD+CR (P<0.05) and OVX+HFD+CR (P<0.001) groups were less than before the CR diet. There was no significant change between sham groups.

**Fig 4:** Effects of CR on TGF-β1 level. Data are expressed as mean ± SEM (n = 4 rats/group). ***P<0.001 *VS*. Sham+SD; ^+++^P<0.001 *VS*. Sham+HFD; ^##^P<0.01 and ^#^P<0.05 *VS*. OVX+SD; ^&&&^P<0.001 *VS*. OVX+HFD; ^†^P<0.05 *VS*. Sham+SD+CR; ^^^P<0.05 *VS*. Sham+HFD+CR. CR: Calorie restriction, HFD: High-fat diet, SD: Standard diet, Sham: Ovary-intact, OVX: Ovariectomy.

### The effect of E2 treatment on TGF-β1 level

The levels of TGF-β1 protein in OVX+SD+E2 and OVX+HFD+E2 groups were lower than OVX+SD+Oil and OVX+HFD+Oil groups (P<0.001). Also, OVX+SD+CR+E2 and OVX+HFD+CR+E2 groups showed less TGF-β1 protein levels than OVX+SD+CR+Oil and OVX+HFD+CR+Oil groups (P<0.05; Fig 5).

**Fig 5:** Effects of E2 administration on TGF-β1 level in OVX rats. Data are expressed as mean ± SEM (n = 7 rats/group). ***P<0.001 and *P<0.05 *VS*. SD+Oil; ^+++^P<0.001 *VS*. HFD+Oil; ^#^P<0.05 *VS*. SD+CR+Oil; ^&^P<0.05 *VS*. HFD+CR+Oil. CR: Calorie restriction, HFD: High-fat diet, SD: Standard diet, OVX: Ovariectomy, E2: 17-β estradiol, Oil: Sesame oil.

### The effect of CR on cardiomyocyte diameter and hydroxyproline content

H&E histological analysis indicated LV cardiomyocyte diameter in the OVX+HFD group was more than the Sham+HFD group (P<0.05, Fig 6A and 6B). On the other hand, in the OVX+HFD+CR group LV cardiomyocyte diameter was less than before the CR diet (P<0.05). There were no significant differences in LV cardiomyocyte diameter with or without CR between the Sham groups. In addition, as shown in Fig 6C, hydroxyproline level has been measured as an evaluation of collagen infiltration in the LV tissue. In the Sham group with or without CR, there was no significant difference between hydroxyproline contents in the LV tissues. However, the OVX+HFD group demonstrated higher hydroxyproline content than the Sham+HFD group (P<0.001). The hydroxyproline level in the OVX+HFD+CR group was lower than in the OVX+HFD group (P<0.05).

**Fig 6:** Effects of CR on LV cardiomyocyte diameter and hydroxyproline content. A) The hematoxylin and eosin stained LV cross sections in experimental groups. B) LV cardiomyocyte diameter bar graphs of experimental groups. Black lines show LV cardiomyocyte diameters in the cell nucleus region. C) Hydroxyproline content in experimental groups (n = 4 hearts/group, ^+++^ P<0.001 *VS*. Sham+HFD; ^###^P<0.001 *VS*. OVX+SD; ^&&&^P<0.001 and ^&^P<0.05 *VS*. OVX+HFD; ^^^^^P<0.001 *VS*. Sham+HFD+CR). CR: Calorie restriction, HFD: High-fat diet, SD: Standard diet, LV: Left ventricular, Sham: Ovary-intact, OVX: Ovariectomy.

### The effect of E2 treatment on cardiomyocyte diameter and hydroxyproline content

Results related to the diameter of LV cardiomyocytes from the hearts of OVX rats treated with E2 are shown in Fig 7A and 7B). OVX+SD+E2 (P<0.05) and OVX+HFD+E2 (P<0.01) groups revealed more reduction in the cardiomyocyte diameter than OVX+SD+Oil and OVX+HFD+Oil groups. Also, LV cardiomyocyte diameter in the HFD+CR+E2 group was less than the HFD+CR+Oil group (P<0.05). Also, after 4 weeks of chronic E2 administration, LV tissue hydroxyproline content was assessed for evaluation of cardiac hypertrophy in OVX animals (Fig 7C). There was a significant reduction in hydroxyproline content in heart tissues of the SD+E2 (P<0.05) and HFD+E2 (P<0.001) groups when compared with the similar oil-treated groups. Also, the administration of E2 in the HFD+CR group led to a decrease in hydroxyproline contents compared with the same oil-treated group (P<0.01).

**Fig 7:** Effect of E2 administration on LV cardiomyocyte diameter and hydroxyproline content in OVX animals. A) The hematoxylin and eosin stained LV cross sections of OVX animals. Black lines show LV cardiomyocyte diameters in the cell nucleus region. B) LV cardiomyocyte diameter bar graphs of OVX rats. C) Hydroxyproline content in heart of OVX rats (n = 4 hearts/group, *P<0.05 *VS*. SD+Oil; ^+++^P<0.001, ^++^P<0.01 and ^+^P<0.05 *VS*. HFD+Oil; ^&&^P<0.01 and ^&^P<0.05 *VS*. HFD+CR+Oil). CR: Calorie restriction, HFD: High-fat diet, SD: Standard diet, LV: Left ventricular, OVX: Ovariectomy, E2: 17-β estradiol, Oil: Sesame oil.

### Effect of CR on *ANP* gene expression

The gene expression analysis performed in the LV of the animals showed that mRNA expression of *ANP* in OVX+SD and OVX+HFD groups was less than in Sham+SD and Sham+HFD groups (P<0.001; Fig 8). In contrast, in OVX+SD+CR and OVX+HFD+CR groups, *ANP* mRNA expression was more than in OVX+SD and OVX+HFD groups (P<0.01). In addition, *ANP* mRNA expression in the OVX+HFD+CR group was lower than the Sham+HFD+CR group (P<0.001). There were no significant changes in *ANP* mRNA expression with or without CR between the sham groups.

**Fig 8:** Effects of CR on ANP mRNA expression in LV tissue. Data are expressed as mean ± SEM (n = 4 hearts/group). ***P<0.001 *VS*. Sham+SD; ^+++^P<0.001 *VS*. Sham+HFD; ^###^P<0.001 and ^##^P<0.01 *VS*. OVX+SD; ^&&^P<0.01 *VS*. OVX+HFD; ^^^^^P<0.001 *VS*. Sham+HFD+CR. CR: Calorie restriction, HFD: High-fat diet, SD: Standard diet, Sham: Ovary-intact, OVX: Ovariectomy, ANP: Atrial natriuretic peptide.

### The effect of E2 on *ANP* gene expression

As seen in Fig 9, OVX+SD+E2 and OVX+HFD+E2 groups showed higher ANP mRNA levels in the LV tissue than OVX+SD+Oil and OVX+HFD+Oil groups (P<0.001). Also, ANP mRNA levels in SD+CR+E2 (P<0.05) and HFD+CR+E2 (P<0.001) groups were more than SD+CR+Oil and HFD+CR+Oil groups.

**Fig 9:** Effect of E2 administration on ANP mRNA expression in the LV of OVX animals. Data are expressed as mean ± SEM (n = 4 hearts/group). ***P<0.001 and *P<0.05 *VS*. SD+Oil; ^+++^P<0.001 and ^+^P<0.05 *VS*. HFD+Oil; ^#^P<0.05 *VS*. SD+CR+Oil; ^&&&^P<0.001 ^&^P<0.05 and *VS*. HFD+CR+Oil. CR: Calorie restriction, HFD: High-fat diet, SD: Standard diet, OVX: Ovariectomy, E2: 17-β estradiol, Oil: Sesame oil.

## Discussion

CR is the most reproducible and potent intervention that delays the undesirable physiologic consequences of chronic diseases such as CVD. In the present study, the protective effects of CR and E2 on obesity-induced cardiac hypertrophy in postmenopausal (OVX) rats were studied. The main findings are that CR and E2 reduced cardiac hypertrophy indices (BW, HW, HW/BW ratio, and LWV), diminished hemodynamic parameters (MAP and HR), TGF-β1 protein level, LV cardiomyocytes diameter, and hydroxyproline concentration, and increased ANP mRNA expression in OVX animals. However, the data showed that E2 injection had similar effects to CR, yet when E2 has associated with CR these effects were more. As mentioned, the findings of the present study have shown that the body weight of the OVX rats which were fed SD or HFD increased. Similar to our study, it has been reported that body weight in OVX animals that were fed with SD or HFD was increased [39]. It is documented that ovariectomy alone causes weight gain, which suggests that estrogen deficiency modifies the body’s metabolic rate, decreasing energy expenditure and causing fat accumulation [40]. In fact, studies have indicated that in postmenopausal conditions, metabolic rate reduction may be accelerated [40]. Also, more energy intake than energy expenditure leads to an increase in fat accumulation and obesity [41].

Obesity is among the main causes of cardiovascular disease, therefore weight loss by diets including CR has been found to improve cardiac function considerably [42, 43]. Although there are various studies on the effect of different diets such as time restriction, and intermittent fasting on the cardiovascular system, the results of these studies show that the CR diet has relative superiority or at least equal compared to other diets on cardiovascular function [44, 45]. Our results showed that CR led to a reduction in body weight in OVX animals that had received both SD and HFD. It has been revealed that CR decreased body weight in OVX animals that received SD and a high triglyceride diet [46]. Also, it has been revealed that severe CR reduced body weight in OVX rats [47]. Furthermore, CR reduced body weight after 6 months in obese patients with type 2 diabetes [48]. On the other hand, chronic E2 treatment like CR diminished body weight in OVX animals that were fed with HFD/SD in our study. It has been indicated that chronic E2 administration decreased the body weight in OVX animals that received SD and HFD [49]. Probable weight loss mechanism(s) caused by E2 includes a reduction in energy intake [50, 51], moderation in fat metabolism [52], effect on adipocytes, and reduced abdominal fat [53].

In another part of this study, we showed that obesity and ovariectomy led to high blood pressure and cardiac hypertrophy in rats characterized by an increment in heart weight, an increase in the cardiomyocyte diameter, and tissue hydroxyproline content. Enhancement in cardiomyocyte diameter and heart tissue hydroxyproline level indicated that hypertrophy in the hearts of ovariectomized obese animals is prominent [1, 54]. This is in line with previous studies that demonstrated high blood pressure and cardiac hypertrophy were induced in ovariectomized obese rats [1, 55]. Moreover, the findings of the present study demonstrated that CR reduced the hydroxyproline level (a substitute marker of collagen), which is one of the cardiac hypertrophy indicators, in OVX rats. In confirmation of these results, it has been shown that alternate-day fasting diminished hydroxyproline content in aged-rat hearts [56]. Studies have represented that the risk of cardiac hypertrophy and high blood pressure in postmenopausal women is more than twice premenopausal women [57, 58], and also cardiac hypertrophy is revealed to be more common in obese postmenopausal subjects [59]. The probable mechanisms include an increment in cardiac output, total blood volume, and the elevated cardiac load imposed on the myocardium [60, 61]. On the other hand, the lack of E2 in menopause situations can elevate hypertension and cardiac hypertrophy [32, 55]. The results of the present study showed that E2 reduced the hydroxyproline level in OVX rats. In this regard, it has been revealed that E2 decreases the hydroxyproline content in OVX animals [62]. It has been reported that E2 reduces collagen synthesis in female hearts and regulates the synthesis of collagen in a sex-related manner [63].

The findings of this study demonstrated that CR decreased MAP, SBP, DBP, HR, and cardiac hypertrophy in OVX animals fed with SD/HFD. It has been documented that CR reduces blood pressure, diastolic dysfunction, and cardiac hypertrophy in humans and rats [64–67]. Moreover, our results showed that E2 therapy, the same as CR reduced these indexes in OVX animals that had received SD or HFD, this indicates that CR could be a suitable substitution for E2 in OVX animals. However, it has been reported that after 6 months of CR, no change was seen in SBP and DBP in obese postmenopausal women [68].

In another part of our study, the possible roles of *ANP* and TGF-β1 in LV cardiac hypertrophy were studied. The results indicated that in OVX animals in both diets (SD/HFD) conditions, the *ANP* gene expression has diminished, and the protein level of TGF-β1 has enhanced. Interestingly, the ovariectomized HFD-fed rats showed lower *ANP* mRNA expression and higher TGF-β1 protein levels than ovariectomized SD-fed rats, demonstrating an additional effect of HFD on *ANP* and TGF-β1 levels. Consistent with these results, it has been demonstrated that cardiac *ANP* gene expression level was low in the ovariectomized rats that were fed SD or HFD [1]. Also, it has been reported that obesity leads to a reduction in cardiac ANP in rodents [69]. While in another study it has been indicated that plasma ANP levels increased in obese type 2 diabetic patients [70]. It is documented that obesity suppresses the biological activity of neuropeptides and leads to an increase in intravascular volume, and cardiac output elevation, and results in cardiac hypertrophy [71]. In addition, TGF-β level has been shown enhance in ovariectomized rats that were fed with HFD [25].

Moreover, our results showed that CR increased the *ANP* mRNA expression and declined the TGF-β1 protein levels in OVX animals that underwent both diet conditions (SD/HFD). Based on the results of the present study and regard to the previous findings, it can be possible to suggest that reduction in *ANP*, and elevation in TGF-β as a secondary inflammatory factor, which are both related to obesity lead to cardiac remodeling and hypertrophy[1, 25]. Also, our data showed that E2 similar to CR enhanced the *ANP* mRNA expression and decreased TGF-β1 protein levels in OVX animals that had received SD or HFD. Evidence has illustrated that estrogen deficiency leads to an elevation of inflammatory factors such as TGF-β [25]. Estrogen also influences the cardiac natriuretic peptide system through stimulation of ANP release, atrial ANP production, and an increase in *ANP* gene expression [72]. Therefore, it seems that ANP is the mediator of estradiol-associated cardiovascular effects [73].

The strengths of the present study were investigating the effects of CR on cardiovascular functional factors such as ANP, TGF-β1, and hydroxyproline content in postmenopausal obese rats. The effects of CR on the process of hemodynamic changes related to the cardiovascular system and histological indices of the ventricular muscle were studied in these animals. Also, cardiac hypertrophy was induced through dietary obesity which is more similar to what happens in humans. In this study, to accelerate menopause induction the animal model of menopause (ovariectomy) was used in young adult rats. Therefore, it is better to use rats with natural menopause to investigate the effects of caloric restriction on cardiac hypertrophy, in future studies.

## Conclusions

Our findings indicate that obesity promotes cardiac hypertrophy and hypertension in ovariectomized animals as an experimental postmenopausal model. Also, our findings indicated that cardiac hypertrophy is associated with a reduction in *ANP* gene expression and elevation of TGF-β1 and hydroxyproline content. On the other hand, the CR diet and chronic E2 treatment prevented cardiac hypertrophy and hypertension in obese OVX animals. Also, the CR diet and E2 therapy increased *ANP* gene expressions and attenuated TGF-β1 protein levels in these animals. In most cases, either the two interventions acted similarly or reinforced each other’s effects. Therefore, CR has a cardiovascular protection effect and may have value as a therapeutic approach for the prevention of cardiac hypertrophy and other cardiovascular complications observed in postmenopausal situations. It is suggested that the effects of this diet on cardiac hypertrophy and hemodynamic parameters be investigated in obese postmenopausal women in future studies.

## Supporting information

S1 Dataset (RAR)
